The article "The Construction and Analysis of a ceRNA Network Related to Salt-Sensitivity Hypertensives" was published in 2022. Journal: Biomed Res Int.

# The Construction and Analysis of a ceRNA Network Related to Salt-Sensitivity Hypertensives

**DOI:** 10.1155/2022/8258351

**Published:** 2022-10-14

**Authors:** Xiu-Juan Liu, Hong-Lin Yin, Yan Li, Hao Hao, Yang Liu, Quan-Lin Zhao

**Affiliations:** ^1^First Clinical Medical College, Shandong University of Traditional Chinese Medicine, Jinan, Shandong 250000, China; ^2^Affiliated Hospital of Shandong University of Traditional Chinese Medicine, Jinan, Shandong 250000, China; ^3^Faculty of Traditional Chinese Medicine, Shandong University of Traditional Chinese Medicine, Jinan, Shandong 250000, China

## Abstract

**Background:**

Salt-sensitivity hypertensives (SSH) are an independent risk factor for cardiovascular disease. However, the mechanism of SSH is not clear. This study is aimed at constructing a competing endogenous RNA (ceRNA) network related to SSH.

**Methods:**

Data sets were collected from the Gene Expression Omnibus database (GEO) to extract data on salt sensitivity RNA of patients with or without hypertensives in GSE135111. Firstly, we analyzed differentially expressed genes (DEGs, log2FC ≥ 0.5 and *P* < 0.05) and differentially expressed lncRNAs (DELs, log2FC ≥1 and *P*<0.05) between SSH and salt-sensitive normotension (SSN). Then, the gene ontology (GO), KEGG pathway enrichment analysis, and PPI network construction of DEGs were performed, and the hub genes in the PPI network by cytoHubba (12 methods) were screened out. Finally, a ceRNA network was constructed based on lncRNA-miRNA-mRNA pairs and hub genes.

**Results:**

163 DEGs and 65 DELs were screened out. The GO and KEGG pathway analyses of DEGs were mainly enriched in metabolism (e.g., insulin secretion and cellular response to glucagon stimulus and peptidyl-tyrosine dephosphorylation,) and plasma membrane signaling (e.g., cell adhesion and chemical synaptic transmission and integral component of membrane). Additionally, a ceRNA network, including 1 mRNA (EGLN3), 2 miRNAs (hsa-miR-17-5p and hsa-miR-20b-5p), and 1 lncRNA (C1orf143) was successfully constructed.

**Conclusions:**

In conclusion, the proposed ceRNA network may help elucidate the regulatory mechanism by which lncRNAs function as ceRNAs and contribute to the pathogenesis of SSH. Importantly, candidate lncRNAs, miRNAs, and mRNAs can be further evaluated as a potential therapeutic targets for SSH.

## 1. Background

Hypertension, one of the most common diseases in humans, is one of the most well-known major risk factors for cardiovascular disease (CVD) and stroke. Accumulating study confirmed a strong relationship between sodium intake and blood pressure. Studies have confirmed that reducing the intake of salt in the diet can effectively reduce blood pressure. However, individuals have different responses to dietary salt. Some people will significantly increase their blood pressure after increasing their dietary salt intake, whereas another part of the population does not show significant changes in blood pressure. This phenomenon is called salt sensitivity [1]. Salt sensitivity is related to multiple factors, including the physiological environment, genetics, and demographic factors. Common demographic factors usually include sex, race, and age. However, the mechanism of salt-sensitivity hypertensives (SSH) is not clear. The mechanism of SSH has become the focus of many researchers.

The article "The Construction and Analysis of a ceRNA Network Related to Salt-Sensitivity Hypertensives" was published in 2022. Journal: Biomed Res Int.

SSH can be defined as elevated blood pressure caused by relatively high salt intake [2]. The mechanism behind the rise in blood pressure caused by increased salt intake is complex. Current studies have found that it is related to an increase in blood volume caused by osmotic pressure, impaired endothelial function, and an imbalance in the regulation of nitric oxide and endothelin [3]. Furthermore, abnormal activation of the renin-angiotensin-aldosterone system, enhanced sympathetic nervous system, insulin resistance, and renal mechanism are also contribute [4]. Genetics, nutritional, and environmental factors are also involved in the development of salt-sensitive hypertension [5]. However, the BP of salt sensitivity differs among individuals. The blood pressure of salt-sensitive people can be divided into SSH and salt-sensitive normotension (SSN). Although both are sensitive to salt, their blood pressure is different. Its internal mechanism has yet to be studied while few people pay attention to their differences.

Herein, we collect hypertension expression data for these three RNAs from the GEO database and construct a competing endogenous RNA (ceRNA) network related to SSH based on the base of DEGs (differentially expressed genes) and DELs (differentially expressed lncRNAs). This is the first study to investigate the ceRNA network related to SSH. After the analysis of DEGs and DELs, we found that some RNAs were tightly related to SSH. The DEGs and pathways predicted in our study may reveal the potential molecular mechanism of SSH. The workflow of this study is shown in Figure 1.

## 2. Methods

### 2.1. Data Collection and Processing

First, the GSE135111 microarray data, including 5 SSH blood samples and 5 SSN blood samples, was downloaded from the GEO database [2]. The microarray data were normalized by R software such as probe identification transformation and log2 transformation. Finally, the normalization data were used for further analysis.

### 2.2. Difference Analysis

In this study, the Limma package [6] was used to identify DEGs (|log2 FC| ≥ 0.5 and *P* value < 0.05), DELs (|log2 FC| ≥ 1 and *P* value < 0.05), and DECs (|log2 FC| ≥ 1 and *P* value <0.05). Then, DEGs and DELs were used in the next analysis.

The article "The Construction and Analysis of a ceRNA Network Related to Salt-Sensitivity Hypertensives" was published in 2022. Journal: Biomed Res Int.

### 2.3. GO and KEGG Pathway Enrichment Analyses of DEGs

Gene ontology (GO) is widely used to annotate genes, gene products, and sequences. KEGG is a comprehensive database for the biological interpretation of genome sequences and other high-throughput data. To represent the characteristics of DEGs, the enrichment analysis of the GO and KEGG pathways of DEGs was performed using a clusterProfiler package with the following criterion: *P* value <0.05.

### 2.4. Construction of the PPI Network and Screening of Hub Genes

To select hub genes related to SSH herein, the DEGs were mapped into PPIs (protein-protein interaction) by the STRING database, and a combined score of >0.4 was set as a threshold value. In addition, nodes with higher degrees of interaction from the PPI network were considered as hub nodes. As everyone knows, cytoHubba [7] is a tool for screening hub genes in the Cytoscape software [8]. Therefore, in this study, the hub gene modules (top 50 genes) were screened out by all 12 methods in Cytoscape software. Only the remaining overlapping genes in all 12 methods were selected as hub genes related to SSH.

### 2.5. Construction of lncRNA-miRNA-mRNA Pairs

As we know, lncRNA-miRNA pairs and miRNA-mRNA pairs can form lncRNA-miRNA-mRNA pairs. miRNA can bind to targeted mRNA to promote the degradation of mRNA, while lncRNA can bind to targeted miRNA to inhibit the degradation of mRNA. Herein, we used ggalluvial R package [9] to construct lncRNA-miRNA-mRNA pairs through miRcode (version 11; http://www.mircode.org/mircode/), miRDB (version 7.0; http://mirdb.org/), miRTarBase (http://mirtarbase.mbc.nctu.edu.tw/index.html), and TargetScan (version 7.2; http://targetscan.org/vert_72/) on the base of DEGs and DELs. miRcode provides “whole transcriptome” human microRNA target predictions based on the comprehensive GENCODE gene annotation, including >10,000 long noncoding RNA genes. Coding genes are also covered, including atypical regions such as 5′UTRs and CDS. miRDB is an online database for miRNA target prediction and functional annotations. All miRDB targets were predicted by a bioinformatics tool, MirTarget, which was developed by analyzing thousands of miRNA-target interactions from high-throughput sequencing experiments. miRTarBase is a database of experimentally validated microRNA targets. TargetScan predicts biological targets of miRNAs by searching for the presence of conserved 8mer, 7mer, and 6mer sites that match the seed region of each miRNA.

The article "The Construction and Analysis of a ceRNA Network Related to Salt-Sensitivity Hypertensives" was published in 2022. Journal: Biomed Res Int.

Firstly, we predicted the lncRNA-miRNA pairs through the miRcode database on the base of DELs. The target genes for these miRNA signatures were then obtained using the miRDB, miRTarBase, and TargetScan databases. Genes present in all three databases were regarded as the target genes for these miRNAs. Comparing predicted target genes with DEGs, only the remaining overlapping genes and their interaction pairs were used for constructing the lncRNA-miRNA-mRNA pairs.

### 2.6. Construction of the ceRNA Network

In this study, the overlapping genes of hub genes and lncRNA-miRNA-mRNA pairs were used as potential key genes related to SSH. In addition, we construct a ceRNA network on hub genes and lncRNA-miRNA-mRNA pairs.

## 3. Results

### 3.1. Identification of DEGs and DELs

After preprocessing and data integration, 163 DEGs (86 upregulated and 77 downregulated), 65 DELs (34 upregulated and 31 downregulated), and 4 DECs (1 upregulated and 3 downregulated) were screened (Figures 2(a) and 2(b)). Herein, the heat map of the lncRNAs, circRNAs, and mRNAs showed that the SSH clustered separately from the paired SSN (Figure 2(c)).

### 3.2. Enrichment Analysis of DEGs

As shown in Table 1 and Figure 3(a). GO and KEGG pathway enrichment analyses of DEGs were mainly enriched in metabolism (e.g., insulin secretion and cellular response to glucagon stimulus and peptidyl-tyrosine dephosphorylation) and plasma membrane signaling (e.g., cell adhesion and chemical synaptic transmission and integral component of membrane).

### 3.3. PPI Network Construction and Screening of Hub Genes

In this study, these DEGs demonstrated significant interactions. A total of 59 nodes of the 163 DEGs were mapped in the PPI network (Figure 3(b)). Four genes (7 ≥Degree ≥4), including *ADCY2*, *TAS2R38*, *TNFSF11*, and *ADCY6*, were located in the center of the PPI network. Additionally, 31 hub genes were selected, including *EGLN3*, *TNFSF11*, and *DPPA4*, and were screened (Table 2 and Figure 4(a)). Furthermore, the top 10 hub genes (radiality method) are shown in Figure 4(b).

### 3.4. Construction of lncRNA-miRNA-mRNA Pairs

Herein, lncRNA-miRNA-mRNA pairs based on DEGs and DELs, including 2 mRNAs (*EGLN3* and *TNFRSF21*), 2 miRNAs (hsa-miR-17-5p and hsa-miR-20b-5p), and 1 lncRNA (C1orf143) was constructed. As shown in Figure 5(a).

### 3.5. Construction of the ceRNA Network

In this study, an overlapping gene (*EGLN3*) between hub genes and lncRNA-miRNA-mRNA pairs was screened out and was identified as a potential key gene related to SSH (Figure 5(b)). Then, based on the potential key genes, a ceRNA network was successfully constructed, including 1 lncRNA (C1orf143), 2 miRNAs (hsa-miR-17-5p and hsa-miR-20b-5p), and 1 mRNA (*EGLN3*).

The article "The Construction and Analysis of a ceRNA Network Related to Salt-Sensitivity Hypertensives" was published in 2022. Journal: Biomed Res Int.

## 4. Discussion

It is generally known that salt sensitivity of blood pressure (SSBP) is an independent risk factor for cardiovascular disease. Although they are both sensitive to salt, their blood pressure is different. The blood pressure of salt-sensitive people can be divided into SSH and salt-sensitive normotension (SSN) [10]. As for SSH, salt sensitivity is related to multiple factors, including physiological environment, genetics, and demographic factors. Common demographic factors generally include gender, race, and age [11]. However, the pathogenic mechanisms of SSBP are still uncertain. Therefore, the mechanism of salt-sensitivity hypertensives (SSH) has become the focus of many researchers.

Nowadays, it has become a popular method for evaluating DEGs through gene expression analysis to explore the causes of diseases [12]. These different genome-wide expression profiling techniques make them more valuable on account of complementary results. In this study, we obtained the analysis of the expression of mRNAs and lncRNAs of whole blood samples from patients with SSH and SSN with active disease and to explored potential RNAs related to SSH by the bioinformatic analysis. Then, we selected 163 DEGs and 65 DELs as our subsequent research object. Furthermore, an enrichment analysis of the GO, KEGG pathway, and the construction of DEG PPI networks were performed, and we found that these 163 genes may participate in the process of SSH through metabolism (e.g., insulin secretion and cell response to glucagon stimulus and tyrosine dephosphorylation) and plasma membrane signaling (e.g., cell adhesion and chemical synaptic transmission and integral component of membrane). This is consistent with previous studies.

In metabolism, such as previous studies have demonstrated that single nucleotide polymorphisms (SNPs) of the sodium-bicarbonate cotransporter gene (*SLC4A5*) are associated with hypertension [13]. Furusho et al. found that mutations of with-no-lysine kinase 1 (*WNK1*) could lead to abnormally increased salt reabsorption and salt-sensitive hypertension [14]. Based on the epidemiological baseline survey, fasting blood glucose was found to be an independent and dose-dependent related factor of blood pressure salt sensitivity [15]. At the same time, it is well known that the ion channel is closely related to SSH. It has been found that there are many pathways mediated phosphorylation of ion channels in the body, including PKA-mediated phosphorylation, PKC-mediated phosphorylation, PI-3 K/PKB and PI-3 K/SGK3 pathway phosphorylation, MAPKs pathway-mediated phosphorylation, and Src channel regulation. However, there are still some signaling pathways that have not yet been reported in the results of our study such as tyrosine dephosphorylation. Tyrosine dephosphorylation is regulated by protein tyrosine phosphatase (PTP). Studies have found that the PTP gene mainly expresses 112 PTP in the human genome. It is not only an indispensable specific regulator in cell signal transduction but also a key signal molecule. It plays a key role in the regulation of different physiological events and is related to many diseases such as metabolism, cardiovascular diseases, cancer, and autoimmune diseases [15].

The article "The Construction and Analysis of a ceRNA Network Related to Salt-Sensitivity Hypertensives" was published in 2022. Journal: Biomed Res Int.

The composition of its catalytic sites determines the sensitivity of dephosphorylation [16]. The same PTP can also be divided into two categories: the receptor tyrosine phosphatase and the nonreceptor tyrosine phosphatase. It is worth noting that the K^+^ channel is closely related to SSH. At the same time, previous articles have reported that K^+^ channels contain multiple tyrosine residues [17]. Some protein enzymes can act on channel protein synthesis and transport to change the phosphorylation state of channel proteins and regulate channel functions. Meanwhile, our results suggest that PTP may be involved in the occurrence of SSH. This gives us great hints. However, whether PTP participates in SSH through the dephosphorylation of K^+^ channel protein remains to be verified by experiments.

In plasma membrane signaling, at present, many types of research are thorough. Such as G-protein coupled receptor signaling pathway and insulin secretion [18]. Note that we constructed an SSH-related ceRNA network, including 1 mRNA (*EGLN3*), 2 miRNAs (hsa-miR-17-5p and hsa-miR-20b-5p), and 1 lncRNA (C1orf143). Among the ceRNA regulatory network, 1 lncRNA (C1orf143) is associated with two miRNAs (hsa-miR-17-5p and hsa-miR-20b-5p), and we proposed that possible competition for C1orf143 binding to hsa-miR-17-5p and hsa-miR-20b-5p influences the downstream regulation of *EGLN3*. However, this requires experimental verification.

*EGLN3* (also named Prolyl-hydroxylase 3, *PHD3*, *HPH1*, and *SM-20*) belongs to the *EGLN* family of prolyl hydroxylases and can catalyze hydroxylation. Studies have shown that *EGLN3* is involved in the metabolism and angiogenesis of oxygen from tumor cells, which in turn affects tumor cell proliferation [19]. However, there is no report about *EGLN3* participating in SSH. It has been reported that *EGLN3* is regulated by miRNA to play a role in different biological processes. However, so far, there has been no research on the *EGLN3* ceRNA network in SSH. What is more, lncRNAs play a significant role in the development of the disease according to many studies. In our study, we found that C1orf143 could lncRNAs play important biological roles by regulating gene expression (a ceRNA network) in SSH. It is worth noting that there is no research report on C1orf143. This is a new gene. Our research results indicate that C1orf143 may play an important role in SSH. This gives us great hints. However, whether C1orf143 is related to SSH still needs further experimental verification.

The article "The Construction and Analysis of a ceRNA Network Related to Salt-Sensitivity Hypertensives" was published in 2022. Journal: Biomed Res Int.

On the whole, based on comprehensive bioinformatics analysis of multiple cohort datasets of SSH and SSN patients, 163 DEGs were identified. The enrichment analysis of DEGs involving related molecules or pathways may deepen our understanding of SSH. Additionally, the SSH-related ceRNA network, including 1 mRNA (EGLN3), 2 miRNAs (hsa-miR-17-5p and hsa-miR-20b-5p), and 1 lncRNA (C1orf143) was successfully constructed. However, some limitations still existed in this research. The main method of our research was bioinformatics technology, a useful tool to understand interactions, pathways, and networks.

In conclusion, these findings could enrich DEG expression profile between SSH and SSN and provide novel information on the occurrence of SSH. Other scientific researchers are expected to verify this at the genetic level.

## Figures and Tables

**Figure 1:** Workflow of this study. Notes: workflow of the study.

**Figure 2:** Difference analysis of mRNAs and lncRNAs. Notes: (a) expression of mRNAs between two sets of samples (SSH vs. SSN). Blue represents the downregulated genes and red represents the upregulated genes, and the names of the 10 genes with the lowest *P* value have been indicated. (b) Expression of lncRNAs between two sets of samples (SSH vs. SSN). Blue represents the downregulated lncRNAs and red represents the upregulated lncRNAs, and the names of the 10 lncRNAs with the lowest *P* value have been indicated. (c) Hierarchical clustering heat map of DEGs (top 57), DELs (65), and DECs (4). Firebrick indicates that the relative expression of mRNAs/lncRNAs/circRNAs were upregulated, navy indicates that the relative expression of mRNAs/lncRNAs/circRNAs were downregulated.

**Figure 3:** Enrichment analysis of DEGs and PPI network construction. Notes: (a) GO and KEGG pathway enrichment analyses of DEGs. (b) PPI network. Red represents upregulated DEGs. Navy blue represents downregulated DEGs, and yellow represents other genes associated with DEGs.

**Figure 4:** Screening of hub genes. Notes: (a) upset plot. The horizontal bar chart shows the number of elements in each collection. The bar chart above represents the number of elements for each intersection and the point represent the relevant set involved. (b) Top 10 hub genes. The redder the color, the stronger their interaction.

The article "The Construction and Analysis of a ceRNA Network Related to Salt-Sensitivity Hypertensives" was published in 2022. Journal: Biomed Res Int.

**Figure 5:** ceRNA network construction. Notes: (a) Sankey diagram for the lncRNA-miRNA-mRNA pairs. Each rectangle represents a mRNA, miRNA, or lncRNA, and the connection degree of each gene is visualized based on the size of the rectangle. (b) Venn diagram of the hub gens and the lncRNA-miRNA-mRNA pairs. The overlapping genes in both represent the potential key genes related to SSH. (c) A ceRNA network. Red represents lncRNAs. Navy blue represents miRNAs. Violet represents mRNAs.

**Table 1:** GO and KEGG pathway enrichment analyses of DEGs.

Category	Term	Count/10	-log10 (*P* value)
BP	Cell adhesion	0.9	1.613392753
	Chemical synaptic transmission	0.6	1.434237533
	Cellular response to glucagon stimulus	0.3	1.428932795
	Peptidyl-tyrosine dephosphorylation	0.4	1.39799905
	Adenylate cyclase-inhibiting G-protein coupled receptor signaling pathway	0.3	1.30207393

CC	Plasma membrane	4.4	1.791142931
	Intrinsic component of plasma membrane	0.3	1.711353914
	Collagen trimer	0.4	1.469118021
	Integral component of membrane	5.1	1.467740938
	Transport vesicle membrane	0.3	1.463466518
	Integral component of plasma membrane	1.8	1.359780188

MF	Transmembrane receptor protein tyrosine phosphatase activity	0.3	2.104180723
	Protein tyrosine phosphatase activity	0.4	1.343534176

PATHWAY	Glutamatergic synapse	0.5	1.867759405
	Insulin secretion	0.4	1.500852037
	Tight junction	0.4	1.475102357

**Table 2:** The first 50 hub genes provided by MCC method.

MCC	Betweenness	BottleNeck	Closeness	ClusteringCoefficient	Degree	DMNC	EcCentricity	EPC	MNC	Radiality	Stress
ADCY6	PSMC4	TNFSF11	ADCY6	HTR1F	ADCY6	HTR1F	GCG	ADCY6	ADCY6	TNFSF11	PSMC4
ADCY2	TNFSF11	PSMC4	TNFSF11	NTPCR	ADCY2	TAS2R38	TNFSF11	ADCY2	ADCY2	PSMC4	TNFSF11
TAS2R38	CSF2	ADCY2	PSMC4	ADCY2	TAS2R38	ADCY6	PSMC4	TAS2R38	HTR1F	CSF2	CSF2
HTR1F	GTSE1	GRIN2A	ADCY2	TAS2R38	TNFSF11	ADCY2	DPPA4	HTR1F	TAS2R38	GTSE1	ADCY6
TNFSF11	ADCY6	KCNT1	CSF2	GCG	KCNT1	GCG	CSF2	GCG	GCG	EGLN3	GTSE1
KCNT1	OBBP2	PTPRB	GTSE1	ADCY6	OBBP2	NTPCR	EGLN3	NTPCR	NTPCR	OCSTAMP	GCG
OBBP2	EGLN3	CSF2	TAS2R38	REP15	CSF2	REP15	GTSE1	TNFSF11	REP15	SPIB	OBBP2
CSF2	GCG	ADCY6	GCG	CLDN24	GCG	CLDN24	OCSTAMP	PSMC4	CLDN24	OBBP2	NTSR1
GCG	NTSR1	GCG	OBBP2	CLDN22	HTR1F	CLDN22	SPIB	CSF2	CLDN22	SDC2	EGLN3
PTPRB	C7orf72	GTSE1	EGLN3	NPPA	PTPRB	NPPA	ADCY6	NTSR1	NPPA	KIF14	ADCY2
PSMC4	KIF14	DPPA4	HTR1F	TNNI3	PSMC4	TNNI3	ADCY2	PTPRR	TNNI3	GAS2L3	TAS2R38
GTSE1	KCNT1	OBBP2	NTPCR	ETV5	GTSE1	ETV5	NTSR1	GTSE1	ETV5	C7orf72	C7orf72
DPPA4	TAS2R38	NTSR1	KIF14	FUT1	DPPA4	FUT1	PTPRB	AKAP5	FUT1	ADCY6	KIF14
FUT1	PLCXD2	EGLN3	OCSTAMP	RASIP1	FUT1	RASIP1	OBBP2	C4BPA	RASIP1	ADCY2	PLCXD2
GRIN2A	ADCY2	FUT1	SPIB	CYYR1	GRIN2A	CYYR1	GAS2L3	EGLN3	CYYR1	GCG	KCNT1
C7orf72	GRIN2A	C7orf72	NTSR1	SLC16A14	C7orf72	SLC16A14	C7orf72	OBBP2	SLC16A14	FCRL1	GRIN2A
NTSR1	PTPRB	SPRY1	C7orf72	ZNRF3	NTSR1	ZNRF3	SDC2	KCNT1	ZNRF3	ZNF577	PTPRB
SPRY1	FUT1	CMTM6	PTPRR	PTPRK	SPRY1	PTPRK	KIF14	PLCXD2	PTPRK	TAS2R38	FUT1
CMTM6	DAO	TAS2R38	AKAP5	GRIN2A	CMTM6	GRIN2A	PTPRR	KIF14	GRIN2A	HTR1F	DAO
EGLN3	SPRY1	DAO	SDC2	FAM124A	EGLN3	FAM124A	AKAP5	PTPRB	FAM124A	ARHGAP44	SPRY1
DAO	CMTM6	KIF14	GAS2L3	GTSF1	DAO	GTSF1	HTR1F	OCSTAMP	GTSF1	NTSR1	CMTM6
KIF14	DPPA4	PLCXD2	PLCXD2	KCNT1	KIF14	KCNT1	TAS2R38	SPIB	KCNT1	NTPCR	DPPA4
PLCXD2	REP15	REP15	FCRL1	TCL1A	PLCXD2	TCL1A	PLCXD2	C7orf72	TCL1A	PTPRR	REP15
NTPCR	CLDN24	CLDN24	ZNF577	OBBP2	NTPCR	OBBP2	NTPCR	GRIN2A	OBBP2	AKAP5	CLDN24
REP15	CLDN22	CLDN22	C4BPA	FCRL1	REP15	FCRL1	GRIN2A	SDC2	FCRL1	CCDC175	CLDN22
CLDN24	NPPA	NPPA	KCNT1	PTPRR	CLDN24	PTPRR	KCNT1	FUT1	PTPRR	C4BPA	NPPA
CLDN22	TNNI3	TNNI3	ARHGAP44	GAS2L3	CLDN22	GAS2L3	FCRL1	SPRY1	GAS2L3	PLCXD2	TNNI3
NPPA	ETV5	ETV5	CCDC175	CCDC175	NPPA	CCDC175	CCDC175	GAS2L3	CCDC175	FAM124A	ETV5
TNNI3	RASIP1	RASIP1	PTPRB	C7orf72	TNNI3	C7orf72	ARHGAP44	CMTM6	C7orf72	KCNT1	RASIP1
ETV5	CYYR1	CYYR1	GRIN2A	ARHGAP44	ETV5	ARHGAP44	ZNF577	DPPA4	ARHGAP44	GRIN2A	CYYR1
RASIP1	SLC16A14	SLC16A14	FUT1	KCNMB3	RASIP1	KCNMB3	CLDN24	ZNF577	KCNMB3	FUT1	SLC16A14
CYYR1	ZNRF3	ZNRF3	FAM124A	C4BPA	CYYR1	C4BPA	CLDN22	DAO	C4BPA	DAO	ZNRF3
SLC16A14	PTPRK	PTPRK	DAO	APOC1	SLC16A14	APOC1	NPPA	FCRL1	APOC1	KCNMB3	PTPRK
ZNRF3	FAM124A	FAM124A	SPRY1	SLC17A4	ZNRF3	SLC17A4	TNNI3	ARHGAP44	SLC17A4	RASIP1	FAM124A
PTPRK	GTSF1	GTSF1	CMTM6	ZNF577	PTPRK	ZNF577	CYYR1	SIGLEC14	ZNF577	PTPRB	GTSF1
FAM124A	TCL1A	TCL1A	DPPA4	SDC2	FAM124A	SDC2	SLC16A14	KCNMB3	SDC2	HOGA1	TCL1A
GTSF1	FCRL1	FCRL1	KCNMB3	CSF2	GTSF1	CSF2	ZNRF3	FAM124A	CSF2	SPRY1	FCRL1
TCL1A	PTPRR	PTPRR	SIGLEC14	AKAP5	TCL1A	AKAP5	PTPRK	CCDC175	AKAP5	CMTM6	PTPRR
FCRL1	GAS2L3	GAS2L3	RASIP1	NTSR1	FCRL1	NTSR1	FAM124A	RASIP1	NTSR1	SIGLEC14	GAS2L3
PTPRR	CCDC175	CCDC175	HOGA1	SPRY1	PTPRR	SPRY1	GTSF1	ETV5	SPRY1	REP15	CCDC175
GAS2L3	ARHGAP44	ARHGAP44	REP15	PTPRB	GAS2L3	PTPRB	TCL1A	REP15	PTPRB	ETV5	ARHGAP44
CCDC175	KCNMB3	KCNMB3	ETV5	SIGLEC14	CCDC175	SIGLEC14	C4BPA	GTSF1	SIGLEC14	DPPA4	KCNMB3
ARHGAP44	C4BPA	C4BPA	GTSF1	CMTM6	ARHGAP44	CMTM6	APOC1	DNMT3B	CMTM6	GTSF1	C4BPA
KCNMB3	APOC1	APOC1	TCL1A	TNFSF11	KCNMB3	TNFSF11	SLC17A4	TCL1A	TNFSF11	TCL1A	APOC1
C4BPA	SLC17A4	SLC17A4	DNMT3B	PSMC4	C4BPA	PSMC4	SPRY1	HOGA1	PSMC4	DNMT3B	SLC17A4
APOC1	ZNF577	ZNF577	CLDN24	EGLN3	APOC1	EGLN3	SIGLEC14	AQP6	EGLN3	CLDN24	ZNF577
SLC17A4	SDC2	SDC2	CLDN22	GTSE1	SLC17A4	GTSE1	CMTM6	PVRL3	GTSE1	CLDN22	SDC2
ZNF577	AKAP5	AKAP5	NPPA	HOGA1	ZNF577	HOGA1	RPL22L1	ZNRF3	HOGA1	NPPA	AKAP5
SDC2	HTR1F	HTR1F	TNNI3	DAO	SDC2	DAO	MRPL15	PTPRK	DAO	TNNI3	HTR1F
AKAP5	SIGLEC14	SIGLEC14	CYYR1	RPL22L1	AKAP5	RPL22L1	DNMT3B	CLDN24	RPL22L1	CYYR1	SIGLEC14

The article "The Construction and Analysis of a ceRNA Network Related to Salt-Sensitivity Hypertensives" was published in 2022. Journal: Biomed Res Int.

## Data Availability

The datasets used during the current study are available from the corresponding authors upon reasonable request (GSE135111).
